The article "Analysis of Rapid Rehabilitation Effect of Children with Severe Viral Encephalitis Based on Continuous Nursing of Omaha System" was retracted in 2023. Reasons: suspected computer-generated content; unreliable results or conclusions; lack of ethics approval or compliance; missing or withdrawn patient consent.

# Analysis of Rapid Rehabilitation Effect of Children with Severe Viral Encephalitis Based on Continuous Nursing of Omaha System

**DOI:** 10.1155/2022/6481697

**Published:** 2022-04-21

**Authors:** Sijia Chang, Yanan Qi, Yingjuan Zhou, Dan Jing

**Affiliations:** Tangshan Maternal and Child Health Care Hospital Department of Pediatrics, Tangshan, Hebei 063000, China

## Abstract

**Objective:**

To establish the Omaha System-based intensive care of children with viral encephalitis, compared with the conventional nursing applied in children with severe viral encephalitis for children with clinical symptoms, motor function, the incidence of complications, and the influence of quality of life, to intensive care of children with viral encephalitis way provide certain scientific basis.

**Methods:**

62 cases of severe viral encephalitis diagnosed and treated in our hospital from X month 20XX to X month 20XX were randomly divided into 31 cases of intervention group and 31 cases of control group. The control group received routine nursing, and the intervention group added Omaha system on the basis of the control group. The recovery time of clinical symptoms and signs, FMA score, disability rate, quality of life, and satisfaction of family members were compared between the two groups.

**Results:**

The recovery time of clinical signs in the intervention group was shorter than that in the control group. Motor function was improved in both groups, but the improvement effect in intervention group was higher than that in control group. The quality of life in both groups was improved 1–3 months after discharge, but the improvement effect in the intervention group was higher than that in the control group. The incidence of physical dysfunction and behavioral abnormalities was low in the pregroup, and the difference between the two groups was statistically significant (*P* < 0.05), but the difference between language impairment and intellectual impairment was not statistically significant (*P* > 0.05).

**Conclusion:**

Omaha system nursing can significantly reduce the recovery time of clinical signs, improve FMA score, reduce disability rate, and improve the quality of life and family satisfaction of children with severe viral encephalitis.

## 1. Introduction

Viral encephalitis is a common disease in pediatric neurology. It is mainly an infectious disease caused by the virus infecting the tissue cells of the central nervous system. It usually causes varying degrees of brain damage [1]. The rise of children's body temperature after onset will lead to serious damage to consciousness, which will pose a threat to children's life. If not treated in time, children will have sequelae such as epilepsy, dyskinesia, and mental retardation, which will have a very serious impact on children's quality of life [2]. In the treatment of children, in addition to routine treatment, reasonable and effective nursing measures can effectively alleviate children's symptoms, reduce the occurrence of complications, and improve the quality of life [3]. Therefore, it is very important to explore the nursing methods suitable for children with severe viral encephalitis and optimize the management of children with severe viral encephalitis. By consulting a large number of relevant literature [4], at present, the research of nursing researchers in China on children with viral encephalitis mainly focuses on rehabilitation nursing. Although relevant nursing interventions can be evaluated after formulation, the lack of standardized language is not conducive to the communication between different nursing and treatment teams. There is a lack of research on the combination of children's health problems with nursing intervention and its effectiveness, and the nursing records are not standardized, so this nursing method cannot be widely used [5].

In the 1970s, the United States created the Omaha system. Omaha system includes a problem classification system, an intervention system, and an effect evaluation system, which is a simplified nursing procedure operating system. At present, it has been widely used in community nursing by health institutions and community service centers in many countries. It is of great significance to standardize nursing records, promote nursing management, and guide practice. Its effectiveness, reliability, and ease of use have been widely recognized by the nursing community [6]. The system has been gradually applied since it was introduced into the Hong Kong Polytechnic University. Although it has been successfully applied to diseases such as hypertension and diabetes, its application is still relatively narrow, and its research on pediatrics is still very small. Although it has been applied to neonates, children with epilepsy and asthma, its applicability and feasibility in pediatrics still need further exploration. At present, there are few reports on the use of this system in children with severe viral encephalitis [7].

The study was based on the evaluation of children's symptoms and the systematic improvement of the quality of life, including the systematic improvement of children's symptoms and the systematic improvement of the quality of life. Thus, it provides a certain scientific basis for the nursing of children with severe viral encephalitis [8]. At the same time, standardized nursing terminology can promote the communication and exchange between medical teams, promote different medical teams to obtain homogeneous training, and realize the continuous, dynamic, and standardized long-term management of children, which has high application value. Omaha System has been widely used abroad, but the application of severe viral encephalitis in China is still rare. On this basis, Omaha System nursing was carried out for children with severe viral encephalitis, and the nursing effect was analyzed.

## 2. Information and Methods

### 2.1. Basic Information

The 62 cases of severe viral encephalitis diagnosed and treated by our hospital in September 20XX to X month 20XX are divided into 62 cases. There were 31 intervention groups and 31 control groups. In the intervention group, there were 16 males and 15 females, with a mean age (9.35 ± 1.29 years) and an average course of illness (6.51 ± 4.36) days; in the control group, there were 18 males and 13 females, with an average age of (9.56 ± 2.12) years. The mean course of the disease is (5.62 ± 4.27) days.

### 2.2. Criteria for Inclusion and Exclusion

#### 2.2.1. Inclusion Criteria

1. Consent to the experiment, and the guardian signs the consent form
2. Meet the diagnostic criteria for severe viral encephalitis
3. The age of the child is 6–13 years old
4. The guardian is familiar with the basic condition of the child in the past three months

#### 2.2.2. Exclusion Criteria

1. Children who are unable to communicate and cooperate normally
2. Children with functional disorders
3. The child's guardian has a history of mental illness
4. Children who are introduced in the middle of the investigation or cannot persist

### 2.3. Research Methodology

#### 2.3.1. Control Group

Routine nursing care is given to the control group, and the nursing staff provides medication guidance to the children's families, conducts health education for the families, informs the families about the relevant knowledge of the children's diseases, and improves the family's cognition. One week after the child was discharged from the hospital, the child was called back to visit the child's diet, activity, and physical condition and gave simple health guidance; after one month, the child was visited at home.

#### 2.3.2. Intervention Group

Increase the Omaha System based on routine care measures. The specific measures are as follows: (1) according to the specific condition of the child's own condition, the Omaha nursing team is established to conduct regular return visits every day before the child's discharge and 1 to 3 months after discharge to investigate and record the child's condition and based on the corresponding treatment measures. (2) The Omaha System was used to evaluate the children in four aspects: social, psychological, physiological, and health. (3) When the nursing problems caused by the child are found in the nursing or follow-up process, corresponding solution measures should be given according to the direction of the care problem, the child's situation. (4) According to the four intervention methods contained in the Omaha System intervention, including treatment procedures, monitoring, health education guidance, and case management, a total of 42 questions and corresponding countermeasures are proposed for each problem to ensure the smooth progress of the nursing plan. (5) The hospital carries out health missions for such diseases in the second week after the child is discharged from the hospital, explaining in detail the knowledge of nutrition, activities, and symptom management, enhancing the family's awareness of the disease and relevant guidance on medication. (6) Notify the family to bring the child to the hospital for follow-up consultation in the third week after the child is discharged from the hospital and conduct a comprehensive examination of the child's physical condition. (7) After the child is discharged from the hospital for 1 month, conduct a family visit to assess the current physical recovery status of the child, give corresponding preventive measures, and continue to follow up with the child's family to ensure the smooth and orderly progress of the nursing plan.

### 2.4. Observing the Indicator

1. Compare the disability of the two groups of children and the recovery time of vital signs
2. The Fugl-Meyer motor function scale is used to assess the child's motor ability, with a full score of 100 points, and the higher the score, the better the motor function.
3. According to the PedsQL^TM^ 4.0 score, comparing the quality of life of the child before discharge and 1–3 months after discharge, the full score is 100 points, and the higher the score, the better the quality of life.
4. The self-made satisfaction evaluation form is used to allow the children's families to assess their satisfaction from five aspects: service attitude, professional skills, health education, psychological counseling, and case management. Out of 100 points, the higher the score, the higher the satisfaction.

### 2.5. Statistical Methods

Use SPSS 23.0 The software performs data processing and measures data to ($\bar{x}\pm s$) represents, rowtTest, counting data using (%) represents, row *x*^2^ inspection *P* < 0.05. The difference is statistically significant.

## 3. Results

### 3.1. Comparison of Basic Information between Children and Families

There were no obvious differences in gender, age, residence status, nutritional status, duration of illness, monthly family income, parental education level, and main caregivers between the two groups, and the two groups were not statistically significant, comparable (*P* > 0.05); for detailed data, see Table 1.

### 3.2. Comparison of the Recovery Time of Vital Signs of the Two Groups of Children

Intervention group: the recovery time of the children's convulsions, impaired consciousness, cranial nerve disorders, and limb disorders was shorter than that of the control group, and the difference between the two groups was obvious and statistically significant (*P* < 0.05); for detailed data, see Table 2.

### 3.3. Comparison of FMA Scores between the Two Groups before and after Care

There was no significant difference in motor function between the two groups before care (*P* > 0.05), and after care, both groups of children had improved motor function; however, in intervention group, the improvement effect of the children was significantly higher than that of the control group, and the difference between the two groups was significant and statistically significant (*P* < 0.05); detailed data are shown in Table 3.

### 3.4. Comparison of Disability of the Two Groups of Children

After nursing, the difference between the two groups of children with language impairment and intellectual disability was not significant, and the two groups were compared. There was no statistical significance (*P* > 0.05), and in the intervention group, the incidence of limb disorders and behavioral abnormalities in children was lower than in the control group, and the difference was significant and statistically significant (*P* < 0.05); detailed data are shown in Table 4.

### 3.5. Comparison of PedsQL^TM^ 4.0 Scores before Discharge and One Month after Discharge

The two groups were compared before and after discharge 1 Months later PedsQL^TM^ 4.0 ScoreTwo groups of children were discharged from the hospital 1. After months, the ratings have increased, but compared to the control group, in the intervention group, the score was higher, with a significant difference between the two groups and a statistically significant *P* < 0.05 [9–11].; detailed data are shown in Table 5.

### 3.6. Comparison of PedsQL^TM^ 4.0 Scores 2 or 3 Months after Discharge from the Hospital in Two Groups

The two groups were analyzed and compared after discharge 2,3 Months later PedsQL^TM^ 4.0 ScoreTwo groups of children were discharged from the hospital 2,3. After several months, the score was significantly improved compared to before discharge, but compared to the control group, in the intervention group, the score was higher, and the difference between the two sets was clearly statistically significant (*P* < 0.05); detailed data are shown in Table 6.

### 3.7. Comparison of Family Satisfaction Scores between the Two Groups

After care, in the intervention group, the scores in service attitude, professional skills, health education, psychological counseling, and case management were higher than those in the control group, and the difference between the two groups was obvious and statistically significant (*P* < 0.05); detailed data are shown in Table 7.

## 4. Discussion

Most children with severe viral encephalitis have acute onset, rapid disease development, and complex disease performance. If children are not treated in time, they will have very serious neurological sequelae and seriously threaten their life and health [12]. The virus dominates the central nervous system and leads to the decrease of motor and neurological function in children. The main symptoms are convulsions, coma, and other symptoms, which seriously affect the prognosis and growth and development of children [13].

At present, there are many effective measures for the treatment of severe viral encephalitis in medicine, and most children can recover their health after reasonable and effective treatment [14]. However, if there is no reasonable cooperation of relevant nursing measures, the treatment effect will not reach the ideal level and even affect the prognosis of the child. At the same time, some children will suffer a certain degree of brain tissue damage during the onset of the disease, resulting in different degrees of sequelae. Although most of the sequelae can be recovered through corresponding treatment, in order to improve the quality of life of the child in the future, effective nursing interventions can be given to help the child return to normal levels. According to the survey [15–17], the incidence of sequelae in children with severe viral encephalitis in China is 50%, and there are about 20% of children who will be disabled. Therefore, the treatment of children is gradually focusing on nursing interventions, and postdischarge care is also very important. The routine mode of care is only a simple guide to discharge considerations, and there is no substantive nursing intervention. Therefore, this study uses the Omaha System intervention to conduct a targeted and in-depth discussion of this problem.

Omaha System is a standardized and comprehensive classification system for nursing practices on the basis of research. It is mainly divided into three interactive and interrelated subsystems: disposal intervention system, problem classification system, and outcome evaluation system [18–20]. The system model is child-centered, and the corresponding care plan is formulated in a targeted and directional manner. The results of this study show that; Intervention group The child's life The recovery time for signs was shorter than in the control group. Both groups of patients had improved motor function, but in the intervention group improvement, the effect was higher than that of the control group. Two groups of children PedsQL^TM^ 4.0 scoring after discharge 1–3 months gradually increase. The improvement effect of the children was higher than that of the control group. Control group dependents total satisfaction score was (71.67 ± 6.59) which was lower than the intervention group (91.25 ± 2.61). After care, in the intervention group, the incidence of limb disorders and behavioral abnormalities in children was low compared to the control group, significantly different, and statistically significant (*P* < 0.05), but there was no significant difference in language impairment and intellectual disability between the two groups, and there was no statistically significant *P* > 0.05 [21]. In recent years, nursing researchers have applied nursing intervention based on Omaha System to children with congenital hydronephrosis, children with severe viral encephalitis, children with neonatal hypoxic-ischemic encephalopathy, and children with epilepsy who underwent nephrostomy, so as to achieve the effect of overall nursing, optimize family continuous care, and reduce long-term adverse events, which is basically consistent with the results of this study. It can be seen that in pediatric disease nursing requiring long-term and effective discharge management, using Omaha System as the basis to formulate continuous nursing strategy can achieve better results.

The Omaha System uses nursing language to guide caregivers to monitor child care problems and provide an effective response plan, effectively intervene from the child's psychological, physiological, and social aspects, and closely integrate child health issues with care plans to improve children's quality of life [22, 23]. While the Omaha System intervenes in nursing problems, according to the development of the child's condition, corresponding nursing measures are given to accelerate the recovery time of the child's vital signs and symptoms, improve the FMA score, and reduce the incidence of disability and the effect of the nursing intervention. Significantly, it also improves the satisfaction of the children's families. Thus, the Omaha systemic care intervention is superior to the usual care intervention [24].

In summary, in the care of children with severe viral encephalitis, the Omaha systemic nursing intervention can significantly reduce the recovery time of the child's vital signs, improve the motor function score, reduce the incidence of disability, and improve the quality of life and family satisfaction.

## Figures and Tables

**Table 1:** Comparison of basic information of children and families.

Project		Control group (*n* = 31)	Intervention group (*n* = 31)	Statistics	*P* value
Gender	Man	18	16	0.179	0.152
	Woman	13	15		
Age (years)		(9.56 ± 2.12)	(9.35 ± 1.29)	0.165	0.321
Whether it is an only child	Be	11 (35.5%)	12 (38.7%)	0.051	
	Not	20 (64.5%)	19 (61.3%)		
Residence status	Rustic	21 (67.7%)	23 (74.2%)	0.452	0.056
	Town	10 (32.3%)	8 (25.8%)		
Nutritional status of the child	Good	29 (93.5%)	30 (96.8%)	0.211	0.061
	Middle	2 (6.5%)	1 (3.2%)		
	Difference	0 (0.00)	0 (0.00)		
Duration of illness (days)	<3	6 (19.4%)	5 (16.1%)	0.351	0.121
	4–6	21 (67.7%)	20 (64.5%)		
	7–10	4 (12.9%)	6 (19.4%)		
Parents' educational attainment	Junior high school and below	6 (19.4%)	5 (16.1%)	1.062	0.332
	High school	17 (54.8%)	18 (58.1%)		
	College degree or above	8 (25.8%)	8 (25.8%)		
Monthly household income (RMB)	<3500	5 (16.1%)	5 (16.1%)	0.261	0.072
	3500–7000	23 (74.2%)	21 (67.7%)		
	>7000	5 (16.1%)	3 (9.7%)		
Primary caregiver	Father	2 (6.5%)	3 (9.7%)	0.513	0.059
	Mother	29 (93.5%)	28 (90.3%)		

**Table 2:** Comparison of recovery time of vital signs in children.

Project	Control group	Intervention group	*T* value	*P* value
Convulsion	5.35 ± 1.17	1.96 ± 0.86	12.362	0.001
Impaired consciousness	5.51 ± 1.31	1.62 ± 0.81	12.213	0.032
Cranial nerve disorders	15.95 ± 3.01	9.77 ± 2.97	9.372	0.000
Limb disorders	16.62 ± 3.37	10.32 ± 2.68	7.133	0.002

**Table 3:** Comparison of FMA scores before and after child care.

Constituencies	Before care	After care	*T* value	*P* value
Control group	49.36 ± 12.61	67.51 ± 21.65	2.892	0.016
Intervention group	49.41 ± 13.01	78.65 ± 22.32	3.976	0.021
*T* value	0.086	2.065		
*P* value	0.126	0.012		

**Table 4:** Comparison of children's disabilities.

Project	Control group	Intervention group	*X* ^2^	*P* value
Language barrier	4 (12.9%)	1 (3.2%)	1.112	0.329
Intellectual disability	3 (9.7%)	1 (3.2%)	0.363	0.156
Limb disorders	7 (22.6%)	1 (3.2%)	3.237	0.001
Abnormal behavior	10 (32.3%)	2 (6.5%)	3.912	0.000

**Table 5:** Comparison of PedsQL^TM^ 4.0 scores before discharge versus 1 month after discharge.

Grouping	Project	Before discharge	Discharged from hospital in January	*T* value	*P* value
Control group	Physiology	46.65 ± 8.12	58.59 ± 6.15	6.135	0.003
Intervention group	Physiology	45.97 ± 8.79	60.12 ± 6.71		
Control group	Emotion	59.51 ± 6.68	71.29 ± 11.09	6.382	0.006
Intervention group	Emotion	60.05 ± 6.96	73.35 ± 2.97		
Control group	Society	56.99 ± 6.12	69.62 ± 9.89	5.992	0.026
Intervention group	Society	57.31 ± 6.27	70.15 ± 8.72		
Control group	Role	39.79 ± 14.62	55.59 ± 15.21	6.761	0.019
Intervention group	Role	40.17 ± 14.77	59.05 ± 14.57		
Control group	Score	49.91 ± 4.38	62.82 ± 5.33	5.562	0.000
Intervention group	Score	51.66 ± 4.32	65.76 ± 5.68		

**Table 6:** Comparison of PedsQL^TM^ 4.0 scores at 2 and 3 months after discharge.

Grouping	Project	Discharged from hospital in February	Discharged from hospital in March	*T* value	*P* value
Control group	Physiology	66.55 ± 5.61	75.36 ± 4.92	5.951	0.015
Intervention group	Physiology	69.97 ± 5.71	78.29 ± 5.01		
Control group	Emotion	77.81 ± 9.36	83.05 ± 8.71	6.057	0.002
Intervention group	Emotion	79.12 ± 8.97	87.13 ± 8.67		
Control group	Society	75.56 ± 8.16	79.68 ± 7.55	5.882	0.000
Intervention group	Society	77.25 ± 8.32	82.06 ± 8.16		
Control group	Role	63.37 ± 9.57	72.33 ± 9.25	6.015	0.031
Intervention group	Role	65.17 ± 8.66	75.06 ± 8.51		
Control group	Score	71.65 ± 5.19	79.15 ± 5.31	5.732	0.006
Intervention group	Score	76.13 ± 5.22	82.12 ± 5.16		

**Table 7:** Comparison of family satisfaction scores in children.

Project	Control group	Intervention group	*T* value	*P* value
Service attitude	15.21 ± 3.37	18.52 ± 2.21	3.872	0.003
Expertise	15.41 ± 4.12	18.92 ± 1.31	4.185	0.021
Health education	14.35 ± 5.36	19.42 ± 0.62	5.026	0.000
Psychological counseling	12.35 ± 4.75	17.38 ± 2.17	5.327	0.000
Case management	13.62 ± 3.57	18.31 ± 1.39	6.296	0.015
Score	71.67 ± 6.59	91.25 ± 2.61	12.52	0.036

## Data Availability

The dataset used in this paper are available from the corresponding author upon request.
